This article has been retracted.

# Machine learning-based e-commerce platform repurchase customer prediction model

**DOI:** 10.1371/journal.pone.0243105

**Published:** 2020-12-03

**Authors:** Cheng-Ju Liu, Tien-Shou Huang, Ping-Tsan Ho, Jui-Chan Huang, Ching-Tang Hsieh

**Affiliations:** 1 Department of Intelligent Commerce, National Kaohsiung University of Science and Technology, Kaohsiung City, Taiwan, China; 2 Department of Leisure and Sport Management, College of Life and Creativity, Cheng Shiu University, Kaohsiung City, Taiwan, China; 3 Yango University, Fuzhou, China; 4 Department of International Business, National Kaohsiung University of Science and Technology, Kaohsiung City, Taiwan, China; University College London, UNITED KINGDOM

## Abstract

In recent years, China's e-commerce industry has developed at a high speed, and the scale of various industries has continued to expand. Service-oriented enterprises such as e-commerce transactions and information technology came into being. This paper analyzes the shortcomings and challenges of traditional online shopping behavior prediction methods, and proposes an online shopping behavior analysis and prediction system. The paper chooses linear model logistic regression and decision tree based XGBoost model. After optimizing the model, it is found that the nonlinear model can make better use of these features and get better prediction results. In this paper, we first combine the single model, and then use the model fusion algorithm to fuse the prediction results of the single model. The purpose is to avoid the accuracy of the linear model easy to fit and the decision tree model over-fitting. The results show that the model constructed by the article has further improvement than the single model. Finally, through two sets of contrast experiments, it is proved that the algorithm selected in this paper can effectively filter the features, which simplifies the complexity of the model to a certain extent and improves the classification accuracy of machine learning. The XGBoost hybrid model based on p/n samples is simpler than a single model. Machine learning models are not easily over-fitting and therefore more robust.

## Introduction

With the rapid development of the Internet, the e-commerce industry has also developed rapidly, and people have increasingly strict requirements for online shopping. For merchants, whether customers can repeat purchases has become a top priority. Channel integration has a strong and positive impact on service quality perception in both online and mobile environments, which further affects transaction-specific satisfaction and cumulative satisfaction. Transaction-specific satisfaction has a positive impact on cumulative satisfaction, which in turn has a positive impact on repurchase intentions. In all dimensions, references and apologies have a greater impact on repurchase intentions through customer satisfaction. By identifying the impact of customer engagement on service interactions, organizations can determine the best role for customers in the service delivery process, enabling more efficient use of organizational resources and improved operational performance.

In addition to the fierce competition in the external market, the inherent problems of e-commerce operators will also cause serious customer losses. The research team at home and abroad conducted in-depth research on customer repurchase. In [1], the author developed and tested a comprehensive online retail ethics model that surveyed sample representatives from various universities in Egypt. The results show that the second-order concept of consumer online ethics (CPORE) includes five ideas and has strong predictive ability to satisfy online consumers. In addition, the authors found that trust and commitment have an important intermediary role in the relationship between CPORE and customer satisfaction. This study developed a comprehensive model of CPORE and empirically tested its multidimensional structure and assessed its impact on consumer satisfaction and buyback intentions through trust and commitment. In [2], the authors found that retaining consumers is critical to multi-channel retailers. The study identified the factors that influence consumer repurchase intentions in an online and mobile retail environment by focusing on the impact of channel integration on the consumer self-regulation process. The authors conducted an empirical test of data collected from consumers of 317 prominent e-retailers in China. The results show that channel integration has a strong and positive impact on service quality perception in both online and mobile environments, which further affects transaction-specific satisfaction and cumulative satisfaction. Transaction-specific satisfaction has a positive impact on cumulative satisfaction, which in turn has a positive impact on repurchase intentions. In [3], the author examines the impact of service failure stage interpretation on customer satisfaction. It attempts to better understand the dynamics of consumer repurchase intentions through the mediation effect of customer satisfaction. The results show that all four aspects of interpretation have a significant partial mediation effect on repurchase intention through customer satisfaction. The results also show that there is no significant relationship between the excuse of service failure and customer satisfaction. In all dimensions, references and apologies have a greater impact on repurchase intentions through customer satisfaction. In [4], the author's study considers the role customers want in an online buying environment. It proposes a model that positions customer-perceived brand innovations as a prerequisite for customer expectations and as a predictor of customer expectations and repeat purchase intentions to meet customer brand satisfaction. The results suggest that product knowledge may have a regulatory effect on the relationship between potential brand innovation and customer expectations. For managers, our research provides useful insights into the ability of online brands to invest in innovative brands to stimulate repeat purchase intentions. In [5], the author designed and tested an empirical model that takes into account the customer's perspective to examine the impact of customer engagement in the service delivery process. The results of the study show that customer engagement has a positive impact on customer satisfaction and emotional commitment through customer relationship values. Emotional commitment is a powerful predictor of repurchase intentions, but does not reveal the relationship between customer satisfaction and repurchase intentions. The findings highlight the role of the client and point to the heuristic value of customer satisfaction and emotional commitment as a consequence of customer engagement. By identifying the impact of customer engagement on service interactions, organizations can determine the best role for customers in the service delivery process, enabling more efficient use of organizational resources and improved operational performance.

Machine learning is a fast, accurate, and highly advanced method. Many experts at home and abroad use it in different fields and have achieved good results. In [6], the author applies the machine learning method to the field of satellite identification economic conditions. The authors demonstrate an accurate, inexpensive, and scalable method for estimating consumer spending and asset wealth based on high-resolution satellite imagery. The authors also show how to train convolutional neural networks to identify image features that can account for up to 75% of local economic changes. The article's model also shows how to apply powerful machine learning techniques with limited training data, which indicates a wide range of potential applications in many fields of science. In [7], the author applied the machine learning method to the health field. Machine learning (ML) is the fastest growing field in computer science, and health informatics is one of the biggest challenges. The goal of ML is to develop algorithms that can be learned and improved over time and can be used for prediction. Most machine learning researchers focus on automated machine learning (aML) and have made great strides in speech recognition, recommendation systems or autonomous vehicles. In the health field, sometimes we encounter a small number of data sets or rare events, and interactive machine learning (iML) may be helpful, rooted in reinforcement learning, preference learning, and active learning. In [8], the author applies machine learning to industrial numerical simulation. The authors propose a data-driven, machine-learning method with physical information for predicting the difference in Reynolds stress in RANS modeling. The machine learning method has observed excellent prediction performance in both cases, proving the advantages of the proposed method. The improvement of the Reynolds stress modeled by RANS by the proposed method is an important step toward predicting turbulence modeling. In [9], the author applies machine learning techniques to the biological health sciences. The use of machine learning and data mining methods in the biological sciences is more important than ever and is critical in intelligently transforming all available information into valuable knowledge. The article predicts and diagnoses complications of diabetes, and systematically reviews the application of machine learning and data mining techniques in the field of diabetes research. Eighty-five percent of the learners used were supervised learning methods, and 15% were unsupervised. In [10], the author applies machine learning to data compression. Inspired by database compression and sparse matrix formats, the authors began the work of value-based compressed linear algebra (CLA), which applied heterogeneous lightweight database compression techniques to matrices and then performed linear algebra operations. The article provides an efficient column compression scheme with a focus on cache operations and an efficient sample-based compression algorithm. Our experiments show that the memory operation performance achieved by CLA is close to the uncompressed case and good compression ratio, which makes it possible to fit a larger data set into the available memory.

This paper analyzes the shortcomings and challenges of traditional online shopping behavior prediction methods, and proposes an online shopping behavior analysis and prediction system. Through the analysis of customer behavior data, the system obtains the customer purchase behavior rules included in the customer, and stores the discovered rule knowledge in the knowledge base. The system is based on the customer's real-time browsing behavior, based on the knowledge in the knowledge base, combined with the customer's personalized attributes, real-time prediction of customer buying behavior trends.

## Method

### E-commerce user behavior prediction model based on decision tree algorithm

Decision trees are a common learning method in machine learning. Good results have been achieved in classification, prediction and rule extraction. The tree structure includes three parts: a root node, a branch node, and a leaf node. It is also a decision node, usually representing a certain attribute of the sample to be classified in the data set. A branch is a different value of the root node, and a leaf node is a possible classification result. The decision tree algorithm divides the training set into relatively pure feature subsets and then recursively builds the decision tree. There are many algorithms based on decision trees. The most widely used is the C4.5 algorithm, which can process not only continuous and discrete attribute data, but also data sets with missing values.

Let S be the training data set, then the information entropy of S is:

$$Entropy(S)=-\sum_{i=1}^{m}p_{i}log_{2}p_{i}$$ (1)

Where pi(i = 1, 2, 3,…, m) is the frequency at which category attributes with m category labels appear in all samples. Suppose A is used to split the data in S. A is discrete and has K different values. Then attribute A divides S into k subsets {S1, S2,…, SK} according to K different values, and the information entropy of attribute A into S is:

$$Entropy_{A}(S)=-\sum_{i=1}^{m}p_{i}log_{2}p_{i}$$ (2)

Where |Si| and |S| are the number of samples contained in Si and S, respectively. Gain(S,A) is the information gain of the attribute A divided into the data set S and the entropy of S minus the entropy of the sample subset after the A division S:

$$Gain(S,A)=Entropy(S)-Entropy_{A}(S)$$ (3)

The C4.5 algorithm introduces split information of attributes to adjust the information gain:

$$SplitE(A)=-\sum_{i=1}^{k}\frac{\left|S_{i}\right|}{\left|S\right|}log_{2}\frac{\left|S_{i}\right|}{\left|S\right|}$$ (4)

For the continuous feature attribute data, the processing of the C4.5 algorithm is performed in the order of increasing attribute values, and the midpoint of each pair of adjacent values is taken as a possible segmentation point, and the left and right partial subsets are segmented according to the segmentation points. The information entropy is used to calculate the minimum value of the information entropy of the data set as the best segmentation point of the attribute, and the minimum information entropy value is used as the attribute entropy of the attribute data set to calculate the subsequent information gain.

### Prediction model of commodity purchase behavior based on XGBoost method

#### Principle of XGBoost algorithm

XGBoost (extreme gradient boosting), also known as extreme gradient boosting algorithm, is a machine learning algorithm that combines decision tree and gradient lifting algorithm. Unlike decision trees generated by algorithms such as ID3 and C4.5, the CART algorithm uses thresholds as the basis for decision tree node splitting, and the threshold is determined by minimizing the mean square error, ie:

$$S=min\left[min_{c_{1}}\sum {\left(y_{i}-c_{1}\right)}^{2}+min_{c_{2}}S{\left(y_{i}-c_{2}\right)}^{2}\right]$$ (5)

After splitting, the left subtree satisfies *R*_1_ = {*x*|*x*≤*S*} and the right subtree satisfies *R*_2_ = {*x*|*x*>*S*}. Since the cart algorithm continuously divides nodes by threshold comparison, the results obtained by the leaf nodes should also be numerical. This determines that the decision tree generated by the cart algorithm is not a "classification tree" but a "regression tree". The bottom layer of the XGBoost algorithm consists of a shopping cart decision tree. It treats these decision trees as the basic "units" of operations and combines them for joint decision making to solve the problem of a single decision tree being over-fitting.

For each sample (Xi, Yi), set its gradient to gm(xi), then the negative gradient direction of model F(xi) is:

$$-g_{m}\left(x_{i}\right)={\left[\frac{\partial L\left(y_{i},F\left(x_{i}\right)\right)}{\partial F\left(x_{i}\right)}\right]}_{F(x)=F_{m-1}(x)}$$ (6)

In order to make Fm(xi) in the direction of -gm(xi), you can use the least squares method to get:

$$\begin{array}{c} a_{m}=argmin\sum_{i=1}^{N}{\left(-g_{m}\left(x_{i}\right)-bh(x;a)\right)}^{2}\\ b_{m}=argmin\sum_{i=1}^{N}L\left(y_{i},F_{m-1}\left(x_{i}\right)+bh\left(x_{i};a_{m}\right)\right) \end{array}$$ (7)

Finally merged into the model: $F_{m}(x)=F_{m-1}(x)+\rho_{m}h\left(x;\alpha_{m}\right)$.

#### Balance positive and negative samples (P/N samples)

When sampling evenly, you need to set the sampling interval k. The size of the interval k directly determines the number of negative samples, while the proportion of negative samples is different. In the sample subset q, the positive sample number is m, the negative sample number is n, and the initial ratio μ of the positive sample to the negative sample is:

$$\mu =\frac{Q_{m}}{Q_{n}}$$ (8)

When the sampling interval is k, the positive and negative sampling rate is μ':

$$\mu^{\prime }=\frac{Q_{m}}{\left(Q_{n}/k\right)}=\frac{k*Q_{m}}{Q_{n}}=k\mu$$ (9)

It can be seen from the above equation that the sampling interval k is linearly positively correlated with the positive and negative sampling rate μ. This means that by finding the k value of the sampling interval, the best positive and negative sampling rate can be obtained.

In order to find a suitable k value, different values are needed to obtain different proportions of positive and negative samples, which are determined based on the post-training score. At the same time, since the cross-validation scores can well express the generalization ability of the model, a 5-fold cross-validation is used in each training to obtain the average of the model scores under different k values. Considering that the positive and negative sample ratios of the original sample subset are about 0, for training data, the positive and negative sample rates should not be too large or too small, so the k value interval is set to 10 to 50 to reduce the running time and the step size is set to 5.

### E-commerce sales forecasting model based on machine learning algorithm and stable volatility model

#### Stable volatility mode

(1) Stable volatility mode

In the sales forecast, the historical sales data can be recorded as: t[m,n], where t(i,j)(i = 1,2,…,n;j = 1,2,…,12) represents the enterprise Sales in the i-th and j-th months. Therefore, the total sales for a year can be recorded as: $t_{i}^{T}=\sum_{j=1}^{12}t_{ij}$. The seasonal factor of the j-th month of the year can be expressed by the following formula: $P_{ij}=t_{ij}/t_{i}^{T},i=1,2,\ldots ,n;j=1,2,\ldots ,12$. If the fluctuation of historical sales data is stable and cyclical, then, month seasonal factors can be more accurately expressed as the average of seasonal factors for the same month each year:

$${\bar{P}}_{J}=\frac{1}{n}\sum_{i=1}^{n}P_{ij},j=1,2,\ldots ,12$$ (10)

#### Support Vector Machine (SVM)

t represents a set of input and output samples (xp, yp). We introduce a support vector machine to solve the regression problem from a simple linear regression problem:

$$y(x)=w^{T}\phi (x)+b$$ (11)

Here we introduce an insensitive error function: $E_{\int }(y(x)-t)=\{\begin{array}{ll} 0, & if\;|y(x)-t|<\int \\ |y(x)-t|-\int , & otherwise \end{array}$, and introduce two relaxation variables $\varepsilon_{n}\geq 0,\;{\hat{\varepsilon }}_{n}\geq 0$, *ε*_*n*_>0 represents the region above the |*y*(*x*)−*t*|<*ϵ*-shaped region y (x), so the error function in the support vector machine regression model can be rewritten as:

$$C\sum_{n=1}^{N}\left(\varepsilon_{n}+{\hat{\varepsilon }}_{n}\right)+\frac{1}{2}\|w{\|}^{2}$$ (12)

The support vector machine plans the prediction problem as a convex programming problem without local minimum values, so there can be a single solution. However, in the optimization process for solving the prediction problem, the artificial neural network may contain multiple local minimum values, so that the final solution is not necessarily the global optimal solution.

#### Artificial neural network

After determining the number of hidden layers, the number of hidden layer units, and the activation function in the artificial neural network model, the information obtained through the training model is stored in the connection of the basic unit, that is, the weight corresponding to each connection. The training process of the artificial neural network is to constantly adjust the parameters *w*_*j*_,*θ*_*j*_,*v*_*j*_,*j* = 1,…,*N* so that the output function y(x) can effectively predict the actual value. The process of training the model uses the following training sets:

$$T=\left\{\left(x^{p},y^{p}\right),x^{p}\in R^{n},y^{p}\in R^{n},p=1,\ldots ,P\right\}$$ (13)

Where (xp, yp) is the input and output set, we denote w as n*N dimension, the vector {*w*_*j*_,*j* = 1,…,*N*} containing the weight of ownership, θ and γ are respectively *θ*_*j*_,*v*_*j*_,*j* = 1,…,*N*-dimensional, including *y*(*x*^*p*^;*w*,*θ*,*v*), j is the input of the given input xp and the neural network. Then, the neural network training process is based on solving the following unconstrained optimization problems:

$$min_{w,q,v}E(w,q,v)=\frac{1}{2}\sum_{p=1}^{P}{\left(y\left(x^{p};w,q,v\right)-y^{p}\right)}^{2}+g_{1}\|w{\|}^{2}+g_{2}\|q{\|}^{2}+g_{3}\|v{\|}^{2}$$ (14)

### E-commerce platform customer repurchase related theoretical basis

#### Customer satisfaction

There are many definitions of the meaning of customer satisfaction: customer satisfaction refers to the evaluation of the customer after the purchase, and is an emotion generated by the customer's subjective judgment and preference during the transaction of the product and service. Customer satisfaction refers to the satisfaction that customers obtain through multiple purchases of products and services; customer satisfaction refers to the customer's perception of the actual acquisition of products and services compared to expected evaluations.

#### Customer repeated purchase intention

The customer's willingness to purchase repeatedly refers to the willingness of the customer to purchase again after purchasing and using the product and service, and is a relatively reliable psychological predictive indicator in the actual repeated purchase behavior of the customer. The final verification results show that there is a positive correlation between the four, but the hierarchical structure of this relationship is different. The two basic factors that determine a customer's willingness to repeat purchases are customer perceived value and conversion cost, and customer satisfaction is customer perception. A derivative value factor ultimately leads to a theoretical model of the customer's willingness to repeat purchases.

#### Customer attitude

Usually, attitude can be divided into three parts, namely, cognition, emotion and behavioral orientation. The cognitive part in the customer's attitude refers to the characteristics of the consumer object that the customer perceives all aspects of the information he has mastered, and the customer assigns the characteristics of the consumer object to different weights according to his own purchasing criteria. The customer attitude affects the customer's evaluation and purchase behavior of the purchased products and services; the emotional part of the customer's attitude is the emotion caused by the customer's positive or negative evaluation process of the purchased product. The emotional part plays the role of up and down linkage, which not only directly affects the cognitive part of the customer's attitude, but also affects the customer's behavioral tendency; the behavioral tendency part mainly refers to the customer's purchase intention in the consumption situation, and the purchase occurs. The premise of the behavior is the reaction to the purchase of the item.

## Experiment

### Data source

According to the 7-day window size, the pre-processed data set is divided into several data subsets every 1-day interval, and then the historical data of each window is obtained through feature extraction and conversion (user id, item id) sample data. According to different windows, it consists of multiple sample subsets. Finally, the "uniform downsampling" method is used to sample the sample subset of each window according to the positive-negative sampling ratio of 1:9, and the obtained positive and negative samples are equalized.

In the obtained sample subset, a subset of the data samples of 10 windows is extracted as the final training data. After sampling, the number of data samples per window is approximately 70,000.

Since the validity of the algorithm selected in this paper needs to be verified, the sample sets of ten windows are divided into two categories: the sample set before feature selection and the sample set after feature selection. The dimensions of the samples were 110 and 56 dimensions, respectively. For convenience of representation, the 10 window sample sets before feature selection are named as training sample set s (1 ≤ i ≤ 10) from small to large, and the sample set after feature selection is named s' (1 ≤ i ≤ 10).

### Experimental environment and tools

Due to the large data set to be processed, the data preprocessing and feature extraction phases in this experiment are based on the server. The server configuration used is shown in Table 1:

**Table 1:** Experimental environment.

Processor	Intel(R) Xeon (R) E5640 2.66GHz*2
RAM	4GB*6
Operating System	Red Hat Enterprise Linux 6.1

The data mining process of this paper uses java language and MySQL for data preprocessing and feature extraction. The logistic regression model uses r language modeling and evaluation models. SVM, decision trees, and XGBoost use Python to build models and optimize models.

### Evaluation method

AUC (area under the curve) is the area under the ROC (Receiver Operating Characteristics) curve. The X-axis of the ROC curve is FPR (false positive rate), and the Y-axis is TPR (true positive rate). The FPR and TPR values can be calculated using the confusion matrix. Here's how to calculate the confusion matrix. For two types of problems, the sample is divided into positive (positive) and negative (negative). When the classification model is classified, there are four cases:

True positive (TP): A positive sample predicted by the model.
False positive (FP): A negative sample predicted by the model as a positive example.
False negative (FN): The positive sample predicted by the model is used as a negative sample.
True negative (TN): A sample predicted to be negative by the model.
Calculate FPR, TPR, and precision based on the confusion matrix:
*FPR* = *FP*/*N*, where n is the number of negative samples;
*TPR* = *TP*/*P*, where p is the number of positive samples;

Accuracy=(TP+TN)/(P+N) (15)

However, in many cases, the roc curve does not clearly indicate which classification algorithm is more efficient, and AUC as a numerical value can intuitively evaluate the quality of the classifier. AUC calculation method such as formula

$$\mathrm{AUC}=\int_{0}^{1}TPRd_{FPR}=\frac{1}{\left(TP+FN)(TN+FP\right)}\int_{0}^{1}TPd_{FP}$$ (16)

AUC is the probability value that the classifier randomly predicts positive and negative samples, and the positive samples are ranked before the negative samples. The larger the AUC value, the better the classification effect.

Usually we use the "F1 value" to measure the accuracy of the prediction of the two types of problems.

$$F1=\frac{2\times \mathrm{Precision}\times \mathrm{Recall}}{\mathrm{Precision}+\mathrm{Recall}}$$ (17)

Among them, the accuracy (precision) refers to the ratio of the number of positive samples with correct classification prediction to the number of positive samples predicted by all classifications. The recall rate refers to the ratio of the positive sample number of the classification prediction to the positive sample number in the original training set.

## Results and discussions

### E-commerce customers repeat purchase forecast results

#### Experimental results of the logistic regression model

Based on the training of the model, the stepwise regression based on the AUC criterion is used to screen the features, and the model is optimized according to the changes of the indicators. The effect of different positive and negative sampling rates on the AUC results of the test set is shown in Fig 1. The accuracy is shown in Table 2.

**Fig 1:** Logistic regression algorithm positive and negative sample ratio on the test set AUC results graph.

**Table 2:** Logistic regression algorithm positive and negative sample proportions on the test set accuracy results table.

Positive and Negative Sample Ratio	1:3	1:5	1:10	1:15
**Accuracy**	0.9355	0.9384	0.9405	0.9421

As the number of training samples increases, the accuracy value increases. The reason is that when the training samples increase, the added samples are mostly negative samples. If the model only learns how to classify negative samples, it will score higher on the test set. The classifier simply classifies all samples as negative samples and also achieves good accuracy. Therefore, here we mainly consider the value of AUC to evaluate the model. By observing the trend of AUC values, it was found that the fluctuation of AUC was not very obvious, but compared with other samples, the 1:3 training model performed best on the test set, and the ratio of positive samples to negative samples was the same. When tilting to a negative sample, the AUC value is lower than the predicted value of the sample ratio of 1:3. This is because as the amount of data increases, the complexity of model training becomes larger and larger, making the results worse. The parameters of the Logistic regression algorithm are obtained by the maximum likelihood estimation method. The purpose of this parameter is to enable the learning model to correctly classify the probability log and maximization of each sample, regardless of whether the sample is a majority or a small number of samples. Class samples, obviously the algorithm is not suitable for category imbalance problems.

#### Model fusion experiment results

The AUC value of the fusion model is iteratively calculated by a large number of artificial weighting values. The logistic regression model was found to be a linear model. The prediction of a single model is not good, and the contribution in the fusion model is not very large. XGBoost is a single model. Not much, XGBoost has a greater impact in training fusion models. The typical weights of several groups are shown in Table 3.

**Table 3:** Manual weighting results.

XGBoost Weight	Logical Regression Weight	Fusion Model AUC Value
0.962	0	0.70231
0.921	0.03	0.69932
0.905	0	0.70015
0.866	0	0.71136

The AUC values of the single model and the fusion model on the test set are shown in Fig 2. The combined model AUC values are nearly 0.15% higher than the optimal model XGBoost in the single model.

**Fig 2:** Single model and fusion model results.

The results of the single model on the training set are trained using the LR algorithm, and the final fusion model is constructed on the test set. The results of constructing the fusion model are shown in Table 4. The AUC values of the fusion models constructed from different single models vary widely. The optimal fusion model is obtained by linear combination of the XGBoost model, but the optimal AUC of the method. This value is the same as the AUC value of the single model XGBoost, with no significant improvement.

**Table 4:** Fusion model for linear model construction AUC results table.

Combined Single Model	Fusion Model AUC Results
XGBoost, Logistic Regression	0.8102
XGBoost	0.7568
Logistic Regression	0.7721

By observing Tables 3 and 4, it is found that the optimal results between the fusion models obtained by the two weighted hybrid prediction methods are not much different, but compared with the two methods, the results of the artificial weighting method are better than the linear model learning weighting method. The reason for this result is that the artificial weighting method is very intuitive to determine the weight value according to the size of the single model AUC value. Only by obtaining the AUC value of the final model to determine whether to increase or decrease the weight, the result is often ideal. The main disadvantage of the linear model is that there is a tendency to overfit, making the model too adaptable to the training set, at the expense of the generalization ability of the unknown test set; too few single models used to construct the fusion model will also lead to the effect of the fusion model. The main reason for the increase is not obvious.

### Analysis of customer demand forecasting model results

To validate the predictive performance of the hybrid model, we compared other widely used sales forecasting methods. Using the same data set as the previous section, we tested the prediction accuracy of the decision tree model, the artificial neural network model, and the single-step support vector machine. Through the training and verification of different models, the decision tree (1,1,1) model is compared with a hidden layer neural network model containing five basic elements, and compared. A support vector machine model that trains historical month sales data values as input vectors.

It can be seen from the prediction results in Fig 3 that the hybrid prediction model based on the stable volatility model and the support vector machine is obviously superior to other prediction models, and the predicted data values are in good agreement with the actual data values. The simple support vector machine model and the artificial neural network model can better capture the nonlinear fluctuation characteristics in the time series than the decision tree model. However, because in some industries, the seasonal fluctuation characteristics of customer demand are very obvious, a hybrid prediction model combining the advantages of stable fluctuation mode and support vector machine can better capture the intrinsic characteristics of data and predict unknown data more accurately.

**Fig 3:** Performance comparison of sales forecasting models in stable volatility mode.

We will further compare the predicted performance curves of the customer model at different subdivision levels, as shown in Fig 4, where the X-axis represents the level of the subdivision. In our experiments, collective marketing and one-to-one marketing each have five advantages. Hierarchical transition, the y-axis represents the average MAPE value, indicating the prediction accuracy. We generated different predictive performance plots for experiments with different parameters. Based on all predicted performance curves, we observed the following results:

**Fig 4:** Comparison of prediction performance at different aggregation levels. (a) High frequency customer set. (b) Low frequency customer set.

The clustering algorithm has good performance on high frequency user sets. As the customer segmentation level continues to be refined, the performance of the predictive model is improved, as shown in Fig 4A. At the same time, this is also the main feature model of the predicted performance curve in this experiment, that is, experiments on most data sets show that customer modeling performance in one-to-one marketing is better than aggregate marketing and segmentation marketing, especially for high frequency customers. Since we have enough data to train a more accurate model, the characteristic pattern of this predictive performance curve is more pronounced.

The clustering algorithm with good performance is on the low frequency user set, and the predicted performance curve is convex, as shown in Fig 4B. This shows that for the low-frequency user set, as the subdivision level is refined, the performance of the prediction model will eventually be affected by data sparsity.

### Prediction of product purchase behavior

#### Algorithm verification

In order to ensure that the f1 value is sufficiently accurate, a ten-fold cross-validation method is adopted, that is, the data of each time window is sequentially used as a test set, and the remaining nine data sets are trained as a training set. At the same time, in order to verify the effectiveness of the algorithm, we use the commonly used machine learning classification algorithm: decision tree, artificial neural network, support vector machine and XGBoost algorithm respectively perform ten cross-validation on the sample set of ten windows, and take the average F1 value. And then use the same method for verification. The sample set after feature selection is named s' for ten-fold cross-validation, and the average F1 value is taken as data comparison. According to the classification algorithm, the average F1 value of the 110-dimensional sample set of the non-selected feature and the average F1 value of the 56-dimensional sample set after the feature selection are classified, and the results are in Fig 5 as follows:

**Fig 5:** Performance comparison of different models before and after feature selection.

It can be seen from the figure that after selecting the SSP algorithm, the F1 value obtained by the different classification algorithms is better than the sample before the feature selection. The improvement of decision tree and support vector machine is not obvious, but the F1 value of artificial neural network and XGBoost algorithm has been significantly improved. Therefore, for the feature selection algorithm, the SSP algorithm has a certain effect on the improvement of the model.

#### Adding positive and negative samples

In order to more intuitively verify the stability of the p/n sample and the XGBoost hybrid model, the F1 values of each training of different models are shown, and the fluctuation amplitude is analyzed. Since the variance ε2 of the decision tree and the logistic regression model is very different from the variance ε2 of the other four models, it is not shown. As Fig 6 shown below:

**Fig 6:** Comparison of different models of F1 oscillation curve.

It can be seen from the above figure that the gbdt and random forest models are significantly behind the prediction accuracy of the p/n samples and the XGBoost and XGBoost models. The p/n samples and the XGBoost and XGBoost models have little difference in the training results for the F1 values. From the perspective of waveform fluctuations, the fluctuations of gbdt and random forest are also larger than the other two models. For P/N samples and XGBoost and XGBoost, the F1 minimum of the XGBoost model training is smaller than the minimum of the P/N sample and the XGBoost model, and the F1 maximum of the XGBoost model training is also slightly larger than the maximum of the P/N sample and the XGBoost model. Therefore, it can be concluded that the waveform vibration interval of the p/n sample and the XGBoost model is smaller than the waveform vibration interval of the XGBoost model. The results also show that the waveform fluctuations of the p/n sample and the XGBoost model are smaller than the overall waveform fluctuation of the XGBoost model.

## Conclusions

This paper analyzes and studies the shortcomings and challenges of traditional online shopping behavior prediction methods, and proposes a network shopping behavior analysis and prediction system. Through the analysis of customer behavior data, the system obtains the customer purchase behavior rules included in the customer, and stores the discovered rule knowledge in the knowledge base. The system is based on the customer's real-time browsing behavior, based on the knowledge in the knowledge base, combined with the customer's personalized attributes, real-time prediction of customer buying behavior trends.

The paper selects linear model logistic regression and decision tree based XGBoost model. After optimizing the model, it is found that the nonlinear model can make better use of these features and get better prediction results. Study the fusion of individual models. In order to avoid the shortcomings of the linear model and the over-fitting of the decision tree model, the model fusion algorithm is used to fuse the prediction results of the single model, and the prediction results are further improved than the single model.

Finally, through two sets of contrast experiments, it is proved that the algorithm selected in this paper can effectively filter the features, which simplifies the complexity of the model to a certain extent and improves the classification accuracy of machine learning. The xgbXGBoost hybrid model based on p/n samples is simpler than a single model. Machine learning models are not easily over-fitting and therefore more robust.
